# Smart Health Monitoring System with Wireless Networks to Detect Kidney Diseases

**DOI:** 10.1155/2022/3564482

**Published:** 2022-10-08

**Authors:** Jyoti Dhanke, Naveen Rathee, M. S. Vinmathi, S. Janu Priya, Shafiqul Abidin, Mikiale Tesfamariam

**Affiliations:** ^1^Department of Engineering Science (Mathematics), Bharati Vidyapeeth's College of Engineering Lavale, Pune 412115, Maharashtra, India; ^2^Department of Electronics and Communication Engineering, IIMT College of Engineering, Greater Noida 201310, Uttar Pradesh, India; ^3^Department of CSE, Panimalar Engineering College, Bangalore Trunk Road, Nazarethpet, Poonamallee, Chennai 600123, Tamilnadu, India; ^4^Department of Electronics and Communication Engineering, K. Ramakrishnan College of Engineering, Samayapuram, Tiruchirappalli, Tamilnadu 621112, India; ^5^Department of Computer Science, Aligarh Muslim University, Aligarh 202002, Uttar Pradesh, India; ^6^Department of Software Engineering, College of Computing and Informatics, Haramaya University, Dire Dawa, Ethiopia

## Abstract

It is essential to change health services from a hospital to a patient-centric platform since medical costs are steadily growing and new illnesses are emerging on a worldwide scale. This study provides an optimal decision support system based on the cloud and Internet of Things (IoT) for identifying Chronic Kidney Disease (CKD) to provide patients with efficient remote healthcare services. To identify the presence of medical data for CKD, the proposed technique uses an algorithm named Improved Simulated Annealing-Root Mean Square -Logistic Regression (ISA-RMS-LR). The four subprocesses that make up the proposed model are a collection of data, preprocessing, feature selection, and classification. The incorporation of Simulated Annealing (SA) during Feature Selection (FS) enhances the ISA-RMS-LR model's classifier outputs. Using the CKD benchmark dataset, the ISA-RMS-LR model's efficacy has been verified. According to the experimental findings, the proposed ISA-RMS-LR model effectively classifies patients with CKD, with high sensitivity at 99.46%, accuracy at 99.26%, Specificity at 98%, *F*-score at 99.63%, and kappa value at 98.29%. The proposed system has many benefits including the fast transmission of medical data to the medical personnel, real-time tracking, and registration condition of the patient through a medical record. Potential enhancement of the performance measures the provider system's hospital capacity and monitoring of a significant number of patients with a concentrated average delay.

## 1. Introduction

An IoT is a key concept that focuses on the modeling and connecting of Internet-linked physical objects using the power of computer systems. Instead of using a certain number of high-powered such as computers, tablet devices, mobile phones, and so on [1, 2], the IoT is largely used for a range of applications using a large number of low-power devices. Such as wrist bands, refrigerators, and umbrellas. Combining IoT with Cloud Computing (CC) is beneficial when it comes to the creation of innovative approaches. An observation model has been built underneath the IoT integration and CC to monitor the state of patients and successfully gather the information, even in distant locations of greater assistance to medical professionals [3]. This model was created to watch the patient's condition. In several situations, the IoT technique is often kept with the assistance of the CC environment to improve efficacy in the deployment of productive resources, data storage, and computational and processing capabilities [4].

The rate at which technological advancements occur is so rapid that almost anything may be connected over the World Wide Web [5]. The phrase IoT pertains to anything that is connected through the Internet. This term describes objects associated with the network and multiple objects connected to process information, and make decisions but also respond to the physical and virtual world [6]. IoT elements including cell phones, engines, sensors, and computing devices generate a significant quantity of data in real-time. The integration of cloud computing with the IoT is the greatest option. CC is indeed the fundamental virtual structure that can be utilized efficiently, and it encompasses many services like servers, networks, and storage [7]. Therefore, the combination of IoT and CC has substantial advantages and benefits in terms of algorithmic resource management, along with the existence and utilization of customizable resources and the usage of these resources as services [8]. There are a significant number of individuals throughout the globe who are afflicted with cardiovascular disease and diabetes may result in a stroke, heart, and kidney failure.

Blood pressure and heart rate sensors, together with an IoT-based cloud and Wi-Fi communications were used in the development of the system for monitoring the health of patients [9]. On the other hand, an actual electrocardiogram-based monitoring system is not included in the system. One such system has been proposed using an Arduino processor, the cloud, an ECG sensor, and a Raspberry [10]. Wi-Fi is used to make the connection to the Internet, and a cloud server receives the data, processes it, and then notifies the appropriate medical personnel in the event of an emergency [11]. It has been proposed that sensors equipment and a heartbeat Fitbit gadget are linked to the CPU through Bluetooth used to create a low-power health monitoring system. It is possible to use a Raspberry Pi as a server to store and process the vital signs of a patient in an emergency and send an alarm to the attending physician [12, 13]. CC is not supported on this system, and the user has a restricted range of motion to work within. Using temperature, pulse rate, ECG, and fall sensors and a Wi-Fi interface to transport the hospital's data to a cloud server, an IoT - based health system was built for real-time monitoring [14]. The system offers to monitor in real-time and makes a medical determination for the patient based on their current data and patient history. On the other hand, the system is not very precise when it comes to making judgments or, in the case of an emergency, alerting medical services [15]. The methods described in the aforementioned body of research provide several difficulties, including those about patient service area, the precision of decision-making, the database, warnings, real-time monitoring from any place, and the dimensions of the device [16].

## 2. Related Works

The purpose of developing and implementing smart watches wireless-based system for health monitoring that reads several vital parameters and then makes a selection based on a methodology that requested the server to contact the necessary person in the event of an emergency [17]. The system gathers information about the patient by employing several sensors and then transmits that information in real-time to a cloud server by way of an Arduino controller. The data is saved inside the cloud using an algorithm that was designed specifically to automatically monitor the health of the patients [18]. The system allows for a degree of adaptability for interaction between patients and the healthcare team using alerts, and it achieves a high level of precision in terms of decision-making [19]. When it comes to delivering medical treatment to a significant number of patients, healthcare institutions and caregivers face a variety of challenges that must be overcome. Because of the explosion in the use of contemporary biomedical sensors and IoT devices, an increasing number of sophisticated medical care and health monitoring systems have been created [20].

The majority of recent research has focused on the early identification of chronic disorders such as CKD, heart disease, and diabetes mellitus. In these studies, numerous factors that may influence chronic disease have been utilized. Despite this, the time complexity and performance of the illness prediction process continue to be significant issues [21]. This is even though all of the critical characteristics that are required for disease prediction are present. When attempting to diagnose CKD, the preliminary components often include a few influencing characteristics. These factors account for the long execution time and low precision of the prediction procedure. In addition to these qualities, however, additional symptoms such as insomnia, chest pain, nausea, and other indicators may also aid in the early diagnosis of probable CKD [22]. CKD stands for chronic kidney disease. Therefore, making use of the approach of feature selection may enhance the overall efficiency of CKD prediction made using a variety of classification strategies.

Then, we apply the important components derived from earlier research for CKD diagnosis in addition to the CKD severity level evaluation, which has not been explored before [23]. This was something that had not been done before. To evaluate the effectiveness of the categorization techniques that were put into practice, the samples needed for this study were taken from a selection of samples [24]. Also, in furthermore to the vital features that have been applied in recent research to predict CKD, several additional clinical symptoms are taken into consideration based on the proposed model [25]. These symptoms significantly contribute to the accuracy with which CKD and its severity degree can be predicted [26]. Therefore, to improve the implementation time and effectiveness of the testing and training process during the classification stage, we pertain to the influencing functionalities based on the clinical observations and experiences of physicians. The findings from earlier studies, provide three groups of crucial characteristics that have an impact on CKD [27]. In addition, if CKD is detected, this model can provide predictions on its subtype. The CKD level is the single most critical predictor in predicting CKD, although it has not been taken into account in any of the prior studies. The entire work done in the past was only devoted to making predictions about the presence of CKD, and the samples were divided into two categories: healthy individuals and CKD patients.

The CC approach is more applicable for finding the basic linear function for NN to provide enough data training [28]. When a model is implemented, the classification procedure focuses on achieving the highest possible level of performance. To solve the problem that occurs in the Neural Network (NN)-CC technique's local optimum, modified techniques of NN-CC have indeed been developed and implemented. The main weights of the neuron connection are responsible for the operation of the NN, and the projected model makes use of the MCS scheme to bring down the overall Root Mean Square Error (RMSE) measurement which is calculated during the NN training process [29]. When contrasted with the NN-CS methodology, the obtained findings indicate that the NN-CC model has achieved an optimal level of function. The overall accuracy of CKD is brought down by the presence of missing values in a dataset. Because the conventional methods are executed during the data preparation stage, the data cleaning task is necessary to complete the work of filling in the missing data and getting rid of the scores that are not useful. It is anticipated that there will be a reevaluation technique used for all stages of CKD in which missing data have been calculated and inserted into the appropriate areas [30]. Even though conventional models are effective, a specialized illness detection system inside a healthcare dataset is still required to guarantee that CKD results are accurate. Within the context of this discussion, the FS task is seen as an essential component of the data categorization process.

This paper presents an ideal IoT and diagnosing chronic kidney disease (CKD) using a cloud-based decision support system, to deliver efficient virtual care to patients. The SA-oriented FS and Root Mean Square Propagation (RMSProp) driven Logistic Regression (LR) model termed ISA-RMS-LR is used by the proposed technique to identify the presence of CKD based on medical data. The proposed model has comprised a group of four different subprocesses, which include data collection, preprocessing, FS, and categorization. The incorporation of SA for FS contributes to the improvement of the classifier results generated by the ISA-RMS-LR model. Using a standard dataset for CKD, the validity of the ISA-RMS-LR model's predictive ability was investigated and confirmed. The results of the experiments suggest that the proposed ISA-RMS-LR model is superior to the methodologies that are being examined in terms of its ability to correctly diagnose and categorize CKD.

## 3. Proposed Model

Figure 1 shows the whole procedure for developing the proposed algorithm of the ISA-RMS-LR model. It depicts the data collecting process that occurs in a variety of ways. Following that, data preparation occurs, and this preprocessed data gets delivered into the ISA-FS model. The ISA-FS approach will choose the optimum subset of attributes, whereas the RMS-LR system will categories them.

In the first step, data is gathered via IoT devices that are connected to patients, a different benchmark healthcare dataset, individual health information, and a hospital administration server. The majority of the medical information provided by IoT devices linked to either a person is essential. A sensor attached to a person, for example, obtains accurate patient records at regular times [31]. CKD data were translated into an acceptable format in three processes. In the beginning, a format transforming operation is performed in which real data are transformed into a .csv file format. Several attribute values together in the dataset, like Absence, Present, and Yes or No, are simultaneously converted to numeric values such as 0 and 1. The median approach would then be used to complete a dataset's missing data.

Figure 2 depicts the general SA technique procedure. The physical aim is for molten material to cool at a minimum pace to assure the process of establishing thermal equilibrium at each temperature. When the temperature approaches absolute zero, the material achieves its ground state, which is composed of relatively low crystalline lattices. When a material solidifies at a temperature below its melting temperature, it forms an unsatisfactory framework that does not consume less energy [32]. In addition, Monte Carlo methods were used to predict the appearance of a material at a particular temperature. A little random disruption to the present state “*l*” of material with energy *S*_1_ created the following state “*n*” with energy *S*_*n*_. As long as *S*_*n*_ is below or equal to *S*_1_, the condition may be considered current. Otherwise, the state has been spent with the following probability.

(1) $$\begin{array}{c} \mathrm{Exp}\left(\frac{\left(S_{1}-S_{n}\right)}{\left(K_{b}T\right)}\right)\text{,} \end{array}$$

where *T*-current temperature; *K*_*b*_-Boltzmann constant.

The Metropolis criteria are given the acceptance rule that was discussed, and the model was used in conjunction with the Metropolis criterion. A state of thermal equilibrium is reached by the material whenever it is heated to any degree because the temperature has indeed been progressively dropping.

(2) $$\begin{array}{c} P_{T}\left(X=1\right)=\mathrm{Exp}{\left(-\frac{S_{1}}{K_{b}T}\right)}_{n}\underset{n}{\sum }\exp\;\frac{\left(-S_{n}\right)}{\left(K_{b}T\right)}\text{,} \end{array}$$

where the sum of the energies of all possible states at temperature “*T*” serves as the denominator in equation (2).

### 3.1. Feature Selection Approach

To diagnose CKD, the proposed method uses the FS methodology. The success of the provided FS technique is contingent on the success of the ISA method which has seen widespread use for combinatorial optimizing tasks. It is presumed that the ISA model is one of the primary search approaches. This will allow the algorithm to find better ways to solve the problem. In this regard, the SA model has the quality of being able to achieve the best solution in contrast to the naive local search algorithm in every given set of conditions.

In most cases, it has been chosen in a completely arbitrary way because it has been a decision to be the best option. The use of the cost function allows for the estimation of the expense of an optimal state in a consecutive manner. When the temperature is unable to match the termination criterion, a solution that is adjacent to the most recent optimum solution is picked, and the cost is evaluated [33]. If the cost of a chosen adjacent solution is lower than or the same as the cost of the most recent optimum solution, then the most recent optimal solution may be swapped out for a new neighbor solution. An arbitrary function within the range has been chosen, even though the cost of nearby solutions is greater when contrasted with the cost of the present ideal solution (0, 1). When we attain this stage, the replacement of the optimum solution is initiated whenever the random value measured against is at its minimum *e*=(cos (*Wn* − cos (*e*=**W**_**a**_))/*T*). After the temperature has been lowered using equation (3), the process is repeated as many times as necessary until the temperature satisfies the termination conditions.

### 3.2. RL-Based Classification Model

A classification task typically generates a presentation that is mapped with datasets of supplied classifications based on current data. Application of the deletion of required data content from a technique for determining the type of data. In the majority of instances, a variable has been required by the LR model for binary classification. This section defines LR approaches by focusing on two types of difficulties. This method's primary objective is to predict the existence of chronic kidney disease, which is typically confirmed using a binary classification methodology. In addition, LR approaches are often used to diagnose illnesses, identify multiple sclerosis, and classify health care data. The function of LR is to predict the presence or absence of CKD. Equation (3) demonstrates that the LR model is mostly reliant upon that linear regression technique:

(3) $$\begin{array}{c} R=\alpha +\beta_{1}i_{1}+\beta_{2}i_{2}+\cdots +\beta_{n}i_{n}\text{.} \end{array}$$

Classification challenges are analogous to continuous-measurement-required linear regression problems. The anticipated value of the categorization model falls between 0 and 1. The outcome is 1 if the numbers are above a specified threshold; otherwise, it is 0. Therefore, the LR parameter sequence falls inside the range [0, 1]. LR indicates that this level employs a sigmoid function. The entire linear model that detects the disease when such a sigmoid function has been applied is a feature.

(4) $$\begin{array}{c} \mathrm{Pr}\;\left(A=+1|B\right)∼\beta .B\;and\;\mathrm{Pr}\left(A=-1|B0=1\;–\;\mathrm{Pr}\;\left(A=+1|Z\right)\right.\text{,}\\ ↓\sigma \left(x\right)=\frac{1}{1+e^{-x}}\in \left[0,1\right]\text{,}\\ \mathrm{Pr}\;\left(A=+1|B\right)∼\sigma \left(\beta .B\right)and,\;\mathrm{Pr}\;\left(A=-1|B\right)=-\mathrm{Pr}\;\left(A=+1|B\right)\text{.} \end{array}$$

Classification is used at both the positive and the negative class levels here. Where “*P*” represents the existence of CKD, “*Q*” indicates the collection of eight elements' independent variables. Each regression model “*Q*” has a coefficient value represented by, which represents the weight. As determined by the LR model, these database values consist of weight values. It provides several linkages between *Q* and *P* for different weights. LR parameters may be altered to get an optimal classification output. At this phase, the RMS model is utilized to choose the LR parameters.

The RMSProp model is based on the construction of such a weighted sum of grades, including such Gradient Descent (GD), using different progression parameters. Consider the scenario and evaluate a cost function made up of contours, with the red dot representing a local optimum. The very first iteration for GD begins at position ‘A' and ends at point ‘B;' Figure 3 shows the other end of an ellipse. The next phase of GD concludes at point 'C.' It reaches the optimum solution in ascending and descending dimensions faster than any prior iteration of GD. Although there is a greater learning value implementation, a lateral oscillation has a significant amplitude and decreases the GD while removing the higher learning value implementation. Vertical oscillations are caused by biases, but the horizontal motion is caused by weight. Vertical oscillation is reduced when the ‘weights' are increased in value and the bias is adjusted. In backward propagation (BP), these parameters d*W* and d*b* are utilized to modify *W*, whereas *b* is a fixed value.

(5) $$\begin{array}{c} W=W–learningrate*dW\text{,}\\ B=B-learningrate*db\text{.} \end{array}$$

RMSprop uses progressively average values of either a squared of d*W* and d*b* rather than the nonepoch-dependent distribution of d*W* and d*b*.

(6) $$\begin{array}{c} SdW=\beta *SdW+\left(1–\beta \right)*\;dW^{2}\text{,}\\ Sdb=\beta *Sdb+\left(1\;–\;\beta \right)*db^{2}\text{,} \end{array}$$

where *β* signifies an alternative hyperparameter that accepts the values 0 and 1, respectively. To compute the new weighted average, the weight from the average of previous values and the square of current values are assumed. In the factors updating process that follows the estimate of upper bound averages, *S*d*W* is quite small and Sd*b* is rather large.

(7) $$\begin{array}{c} W=W–learning\;rate*\frac{dW}{\sqrt{SdW}}\text{,}\\ b=b–learning\;rate*\frac{dW}{\sqrt{Sdb}}\text{.} \end{array}$$

### 3.3. Performance Validation

The effectiveness of the provided paradigm is validated by a comprehensive comparison with current practices. The proposed simulation was performed using MATLAB software. The number of Maximum iterations is set to 20, the Maximum Subiterations number is set to 5, and Initial Temp T0 is set to 10, with Temp. Reduction Speed alpha is set to 0.99.  Table 1 depicts the dataset's overview and its accessible elements. The CKD dataset has a total of 400 occurrences with 24 characteristics. 250 occurrences are categorized as having chronic kidney disease (CKD), whereas the remaining 150 examples are designated as not having CKD.

## 4. Results and Discussion

The results of applying FS models to the CKD dataset are shown in Table 2, which can be found here. The optimum cost analysis of such SA-FS model that was supplied may be seen shown in Figure 4. With the best cost of 0.79, the table values proposed that perhaps the CFS model produced worse FS outcomes. In addition, it is shown that the best cost of the Principal Component Analysis technique is 0.04670, which is somewhat less than CFS but not significantly lower than competing models. The GA-FS and PSO-FS models have surpassed their predecessors and achieved almost equal best costs around 0.04640 and 0.04746, respectively. However, the proposed SA-FS model has selected just the thirteen qualities with the optimum cost, which is 0.01105. This lowest possible cost supplied by the SA-FS model ensured its greater performance in comparison to its predecessors.

Figure 5 depicts the various confusion matrices resulting from either the implementation of RMS-LR technology without FS at various epoch counts. The RMS-LR model has identified 182 cases as active and 150 instances as missing, as shown by the epoch count of 400. Likewise, for the epoch value of 800, the RMS-LR algorithm has categorized 117 cases as current and 150 occurrences as missing. Similarly, under the epoch value of 1200, the RMS-LR algorithm has identified 237 occurrences as present and 147 as missing. Concurrently, the RMS-LR algorithm has identified 242 cases as active and 146 occurrences as missing under the 2000 epoch count.

Figure 6 depicts several confusion matrices resulting from implementing ISA-RMS-LR using FS at varied epoch counts. Using such a different epoch count of 400 indicates that the ISA-RMS-LR method has identified 243 occurrences as present and 145 instances as missing in a collection. Similarly, a count of 800 epochs demonstrates that the ISA-RMS-LR system classifies 243 cases as present and 145 instances as missing. By this, it is seen that, under the epoch count of 1600, the ISA-RMS-LR method has categorized 247 occurrences that were present and 146 instances were absent. The ISA-RMS-LR algorithm has categorized 246 cases as present and 146 instances are absent under the 2000 epoch count.

After evaluating the classifier results provided by an ISA-RMS-LR system under various epoch counts, it was determined that perhaps the ISA-RMS-LR model may provide the most precise classification performance when the epoch count is between 1600 and 2000.  Figure 7 demonstrates that in this specific round, the ISA-RMS-LR algorithm classifies 247 cases as present and 146 instances as absent.

Figure 8 illustrates the accuracy of the RMS-LR and ISA-RMS-LR models concerning the 2000 epoch data. The ISA-RMS-LR produces more accuracy than the RMS-LR method. The precision of both proposed models increases as the number of epochs increases, reaching a peak at 2000 epochs.  Figure 9 illustrates the loss curves for the RMS-LR with ISA-RMS-LR algorithms for varied numbers of 2000 epochs. It has been demonstrated that the ISA-RMS-LR model produces a lower loss rate than the RMSPO-LR model. The real loss of the proposed models starts to decrease as the number of epochs increases and becomes constant around 2000 epochs. The addition of an SA-based FS procedure dramatically reduces the loss graph, as seen.

The outcomes of the ISA-RMS-LR model to those of current models for a variety of metrics compare in Table 3.  Figure 10 presented a comparative examination of the sensitivity and specificity of the ISA-RSM-LR model's findings. In addition, it is discovered that the D-ACO yields successful outcomes with sensitivity and specificity values around 86.00% and 83.35%, respectively. Upon continuation, the DT model yields a somewhat tolerable performance using sensitivity and precision values of 91.38% and 88.28%, respectively. Similarly, the MLP model must achieve a classifier with sensitivity and precision values of around 93.30% and 93.86%, respectively. Simultaneously, the FNC model has shown consistent results, having sensitivity and accuracy values around 85.69% and 85.75%, respectively. The RMS-LR model has generated an effective classifier having sensitivity and accuracy values of around 98.35 percent and 97.09 percent, respectively. The maximal sensitivity and specificity values for the proposed ISA-RMS-LR models are 99.46% and 98%, respectively. In addition, it is shown that the LR has a significantly superior Kappa value of around 74.60%. In contrast, it is obvious that perhaps the XGBoost algorithm has achieved the same Kappa value at 75.42 percent. In addition, the PSO model beat current frameworks with a 68% higher Kappa value. In addition, ACO prefers to provide effective outcomes with a Kappa value of around 73.06%. However, with Kappa values of around 79.37%, the DT model produced slightly reasonable results. With Kappa values of 84.78 percent, the MLP model also achieves good classifier performance. Likewise, the FNC structure has shown consistency with a Kappa value of around 91.87 percent. Concurrently, it is obvious that the D-ACO approach produced a Kappa value that is even higher, 88.33%. With both a Kappa value of 94.63 percent, the RMSPO-LR system is projected to provide competitive classification results. Therefore, the proposed ISA-RMS-LR method has produced results with a superior Kappa value of 93.26 percent. By evaluating the previous tables and graphs, it is determined that the RMSPO-LR model is a suitable medical diagnosis for CKD and may be utilized in real-time.

## 5. Conclusion

Using the ISA-RMS-LR model, this research assessed the optimal IoT and cloud-based decision support method for diagnosing CKD. Initially, the data collecting method captures the patient's information via medical devices. The gathered data are then preprocessed in preparation for future processing. The SA-FS method is then executed, and a subset of characteristics is provided to RMS-LR-based classifiers. The proposed classifier correctly identified the existence of CKD. The results of a detailed experimental investigation are verified using a benchmark dataset of CKD. The simulation results are reviewed for a range of epoch counts. According to the experimental findings, the proposed ISA-RMS-LR model effectively classifies patients with CKD, with high sensitivity at 99.46%, accuracy at 99.26%, Specificity at 98%, *F*-score at 99.63%, and kappa value at 98.29%. The obtained findings demonstrated the improved classification performance in comparison to the techniques evaluated. Clustering approaches may be used to enhance the performance of both the ISA-RMS-LR CKD diagnostic model as part of our future research. The framework intends to provide a complete patient history at home and around the world where the worldwide cloud server is frequently used, allowing the patient to easily access but also track health care providers from any location by logging through into platform, transferring past data, and accessing the web page data.

## Figures and Tables

**Figure 1:** Proposed CKD system.

**Figure 2:** Simulated annealing model.

**Figure 3:** General RMSProp progress model.

**Figure 4:** Comprehensive cost estimate of the ISA-FS technique.

**Figure 5:** Confusion matrix for RMS-LR from 2000 Epoch FS.

**Figure 6:** Confusion matrix of proposed system 2000 Epochs.

**Figure 7:** Confusion matrix for 1600th iteration.

**Figure 8:** (a) RMSPO-LR accuracy graph with 2000 Epochs (b) ISA-RMS-LR accuracy graph with 2000 Epochs.

**Figure 9:** (a) RMS-LR Loss Graph with 2000 Epochs (b) ISA-RMS-LR Loss Graph with 2000 Epochs value.

**Figure 10:** Performance measures.

**Algorithm 1:** ISA-Based Feature Selection.

**Table 1:** Dataset description.

Description	Value
Instances count	535
Features count	28
Class count	3
Percentage of positive samples	72.56%
Percentage of negative samples	37.52%
Data source	Own data from UCI data repository

**Table 2:** Analysis with CKD detection feature selection methodology results.

Methods	Best cost	Selected features
Proposed system	0.01054	7, 14,8,10,20,6,5,13,4,2,3
PSO-FS	0.03657	15,13,24,23,12,20,12,7,19,2,8,2,14,4,1,5,18,17
GA-FS	0.03440	15,23,12,8,13,16,21,19,2,14,24,17,13,5,3,9,3,20
PCA	0.04570	1,2,3,4,5,6,7,8,9,10,11,12,13,14,15,16,17,18,19

**Table 3:** Proposed Method using the Performance Evaluation of CKD.

Classifiers	Performance measures				
	Sensitivity (%)	Specificity (%)	Accuracy (%)	F-score (%)	Kappa (%)
ISA-RMS-LR	99.46	98	99.26	99.63	98.29
RMSPO-LR	98.35	94.86	97.09	97.59	93.63
FNC	85.69	85.88	85.75	86.64	88.88
D-ACO	86.00	83.35	85.00	86.03	89.34

## Data Availability

No data were used to support this study.
